The article "Assessing Nigrostriatal Dopaminergic Pathways via 123I-FP-CIT SPECT in Dementia With Lewy Bodies in a Psychiatric Patient Cohort" was published in 2021. Journal: Front Aging Neurosci.

# Assessing Nigrostriatal Dopaminergic Pathways *via* 123I-FP-CIT SPECT in Dementia With Lewy Bodies in a Psychiatric Patient Cohort

**DOI:** 10.3389/fnagi.2021.672956

**Published:** 2021-06-21

**Authors:** Niels Hansen, Claudia Lange, Charles Timäus, Jens Wiltfang, Caroline Bouter

**Affiliations:** ^1^Department of Psychiatry and Psychotherapy, University Medical Center Göttingen, Göttingen, Germany; ^2^German Center for Neurodegenerative Diseases (DZNE), Göttingen, Germany; ^3^Neurosciences and Signaling Group, Department of Medical Sciences, Institute of Biomedicine (iBiMED), University of Aveiro, Aveiro, Portugal; ^4^Department of Nuclear Medicine, University Medical Center Göttingen, Göttingen, Germany

**Keywords:** dementia with Lewy bodies, 123I-FP-CIT SPECT, psychiatry, prodromal dementia with Lewy bodies, psychopathology

## Abstract

**Background:**

(123)-I-2-ß-carbomethoxy-3ß-(4-iodophenyl)-N-(3-fluoropropyl) nortro- pane single photon emission computed tomography (123I-FP-CIT SPECT) was validated to distinguish Alzheimer’s dementia from dementia with Lewy Bodies (DLB) by European medical agencies. Little evidence exists that validates 123 I-FP-CIT SPECT as a supplementary method to diagnose probable DLB in a psychiatric cohort of patients with psychiatric symptomatology and suspected DLB. We aim to elucidate differences in the clinical phenotype of DLB between those patients with and those without a positive 123 I-FP-CIT SPECT indicating a nigrostriatal deficit.

**Methods:**

To investigate this, we included 67 patients from the Department of Psychiatry and Psychotherapy at University Medical Center Göttingen (UMG) in our study who had undergone 123I-FP-CIT SPECT in the Department of Nuclear Medicine (UMG) by evaluating their patient files.

**Results:**

55% with a positive-123I-FP-CIT SPECT and probable DLB after the 123I-FP-CIT SPECT exhibited psychiatric features. The number of probable DLB patients in those exhibiting psychiatric symptoms was higher post-123I-FP-CIT SPECT than pre-123I-FP-CIT SPECT assessed cross-sectionally over a 6-year period (*p* < 0.05). In addition, prodromal DLB and prodromal DLB patients with a psychiatric-phenotype yielded higher numbers post-123I-FP-CIT SPECT than pre-123I-FP-CIT SPECT (*p* < 0.05). Furthermore, we discovered no phenotypical differences between those DLB patients with a positive and those with a negative 123I-FP-CIT SPECT. 123I-FP-CIT SPECT-positive DLB patients in our psychiatric cohort revealed a psychiatric onset more often (52%); DLB was less often characterized by an MCI onset (26%) (*p* < 0.005).

**Conclusions:**

Our findings support 123I-FP-CIT SPECT as an adjuvant tool for improving the diagnosis of probable DLB and prodromal DLB in a cohort of psychiatric patients with often concomitant psychiatric symptomatology. The psychiatric-onset is more frequent than an MCI-onset in DLB patients presenting nigrostriatal dysfunction, giving us an indication of the relevance of deep clinical phenotyping in memory clinics that includes the assessment of psychopathology.

The article "Assessing Nigrostriatal Dopaminergic Pathways via 123I-FP-CIT SPECT in Dementia With Lewy Bodies in a Psychiatric Patient Cohort" was published in 2021. Journal: Front Aging Neurosci.

## Introduction

Dementia with Lewy bodies (DLB) is a frequent neurodegenerative dementia occurring in about 8% of all dementia patients (Walker et al., 2015). The proportion of DLB patients might be underestimated, as a neuropathological study showed in patients with dementia, 41% revealed Lewy body pathology (Wakisaka et al., 2003). However, Lewy body pathology has also been frequently detected coincidentally post-mortem in patients without dementia (Wakisaka et al., 2003). As these studies reveal a mismatch between diagnosis during life and post-mortem, we should be aiming to improve the early diagnosis of DLB. An DLB diagnosis is often impeded by a severe psychiatric presentation (Borda et al., 2020; McKeith et al., 2020; Segers et al., 2020). Visual hallucinations as a psychiatric symptom are one of DLB’s core clinical features associated with locating Lewy-body pathology (Sakai et al., 2019) and is incompatible with other psychiatric disorders such as schizophrenia. Other core clinical features comprise parkinsonism, fluctuating attention, and cognition, and rapid eye movement (REM) sleep behavioral disorder (McKeith et al., 2017). In addition to the disease’s core clinical features, supportive criteria for diagnosing DLB are psychiatric features like delusions, other hallucinations, apathy, fear, or depression according to McKeith et al. (2017). Suspected DLB patients exhibit a neuropsychological profile suggesting Lewy Body pathology, such as visuospatial deficits or attentional executive dysfunction with relatively intact episodic memory function. Though some DLB patients also show memory deficits (Coughlin et al., 2020), which makes it difficult to distinguish them from patients with Alzheimer dementia. To diagnose DLB according to McKeith’s criteria (McKeith et al., 2017), the patients must display a progressive dementia interfering with daily living activities. Possible DLB is fulfilled if one core clinical feature is present. Potential DLB can be diagnosed if no core clinical feature is identified, but if the indicative biomarker (123)-I-2-ß-carbomethoxy-3ß-(4-iodophenyl)-N-(3-fluoropropyl) nortropane single photon emission computed tomography (123I-FP-CIT SPECT) reveals a uni-or bilateral nigrostriatal deficit, it is a positive result. Probable DLB can be diagnosed when these conditions are fulfilled: (1) two core clinical features are present or (2) one core clinical feature is present and the 123I-FP-CIT SPECT is positive. To diagnose prodromal DLB, McKeith’s criteria (McKeith et al., 2020) served to differentiate between an onset with psychiatric symptoms, onset with mild cognitive impairment (MCI), or onset with delirium. Supporting psychiatric features can lead to a possible DLB diagnosis if the 123I-FP-CIT SPECT is positive. 123I-FP-CIT SPECT reveals dopaminergic nigrostriatal neuronal cell loss (Palermo and Ceravolo, 2019) typical for DLB. It is known to differentiate between DLB and other forms of dementia (Brigo et al., 2015). 123I-FP-CIT SPECT is known as an indicative biomarker for diagnosing DLB, and is thus used to provide supplemental evidence according to McKeith’s criteria (McKeith et al., 2017). It facilitates the diagnosis of possible or probable DLB. Furthermore, it might prove worthy when deciding on the subsequent therapy for DLB in patients with suspected DLB (Kemp et al., 2011; McCleery et al., 2015; McKeith et al., 2017) or probable DLB (McKeith et al., 2017). However, there is much less data on DLB patients who present in psychiatric institutions than there is on most patients presenting in a neurology department or a memory clinic’s outpatient unit. DLB is known to potentially begin with psychiatric symptoms, or even depict a concomitant or predominant psychiatric symptomatology (Ballard et al., 2004; Chiu et al., 2017; Fujishiro et al., 2018). The aim of this study is to confirm whether 123I-FP-CIT SPECT has an additive value for diagnosing DLB in a homogeneous cohort of psychiatric patients often presenting with additional or pure psychiatric symptomatology with suspected DLB, namely (1) possible DLB and (2) prodromal DLB patients, or (3) patients with suspected DLB following neuropsychological investigation. Furthermore, we aim to elucidate differences in actual phenotype between DLB patients with psychiatric- vs. mild cognitive-onset of symptoms diagnosed as DLB *via* 123I-FP-CIT SPECT. Furthermore, we want to assess any differences in the neuropsychological and clinical phenotypes of patients with a positive 123I-FP-CIT SPECT vs. those with a negative 123I-FP-CIT SPECT.

The article "Assessing Nigrostriatal Dopaminergic Pathways via 123I-FP-CIT SPECT in Dementia With Lewy Bodies in a Psychiatric Patient Cohort" was published in 2021. Journal: Front Aging Neurosci.

## Materials and Methods

We conducted a retrospective and observational study in 67 patients from a base cohort of 825 patients that received a 123I-FP-CIT SPECT in the Department of Nuclear Medicine of the UMG with suspected DLB who were examined in the Department of Psychiatry of the University Medical Center Göttingen (UMG). Probable and possible DLB patients were diagnosed in accordance with the McKeith criteria (McKeith et al., 2017), as was a prodromal DLB diagnosis (McKeith et al., 2020). All patients underwent 123I-FP-CIT SPECTs in the Department of Nuclear Medicine University Medical Center Göttingen.

### 123I-FP-CIT SPECT

All patients underwent 123I-FP-CIT SPECTs in the Department of Nuclear Medicine at the University Medical Center Göttingen. They underwent 123I-FP-CIT SPECT to determine the functional integrity of nigrostriatal pathways. SPECT images of the brain were taken 3.5 h after an intravenous injection of approximately 185 MBq of 123I-FP-CIT. Images were taken with a double-headed GE Discovery 630 NM SPECT camera (GE Healthcare, Chicago, IL, United States). A 128 × 128 matrix at an energy setting of 159 keV ± 10%. Images were reconstructed *via* the ordered subset expectation maximization (OSEM) algorithm. OSEM consists of 5 iterations, 10 subcategories as well as a Butterworth filter. We employed Chang’s attenuation correction technique. Image analysis was done visually and semi-quantitatively using GE DaTQuant (GE Healthcare, Chicago, IL, United States). 123I-FP-CIT-SPECT images were visually rated abnormal if: (1) tracer uptake was asymmetric between the hemispheres with a marked reduction in one of the putamen, (2) was reduced bilaterally within the putamen, or (3) was bilaterally absent. Furthermore, semi-quantitative analysis of striatal uptake was done with DaTQuant and the left and right striata-to-background ratios (SBRs) were calculated using a background region of interest over the occipital lobe representing cortical background. The lowest SBR between right and left striata was used for further analysis as described and applied in clinical practice (Tossici-Bolt et al., 2006). All drugs were discontinued that may influence 123I-FP-CIT binding.

### Clinical and Neuropsychological Phenotyping of Patients

All patients received neuropsychological testing and clinical phenotyping. The time interval between neuropsychological testing and the 123-FP-CIT SPECT investigation was at most 6 months. Neuropsychological testing to determine a mild cognitive decline progressing to dementia was carried out using the Diagnostic and Statistical Manual of Mental Disorders (5th edition: DSM V). Neuropsychological testing was done to assess patients’ performance in cognitive domains via a detailed neuropsychological test battery including the Consortium to Establish a Registry for Alzheimer’s Disease (CERAD)-Plus. Mild cognitive impairment (MCI) was defined as a neuropsychological performance below -1 to -2 fold of the standard deviation in one or more cognitive domains. The clinical features and supportive biomarkers were retrospectively evaluated by relying on electronic patient records. The following terms (clinical features and biomarkers) were assessed applying a dichotomous score that indicates whether the symptom is present (score = 1) or not (score = 0): fluctuating cognition, REM sleep behavioral disorder, repetitive hallucinations, parkinsonism, neuroleptic hypersensitivity, postural instability, falls, transient episodes of unresponsiveness, syncopes, severe autonomic dysfunction, hypersomnia, hyposmia, parkinsonism, hallucinations in other modalities, delusions, apathy, anxiety, depression and supportive biomarkers [temporal preservation and electroencephalography (EEG) slowing]. Hyposmia was assessed *via* the patient history documented in patient files. The same was done for RBD patients who had not undergone polysomnography, but whose prior diagnosis or related facts in their patient history suggested RBD. We excluded patients from our cohort who exhibited any other reasons for cognitive or motor impairment such as Alzheimer’s disease, Parkinson’s disease dementia, Parkinson’s disease, or other neurodegenerative disorders such as multiple system atrophy or progressive supranuclear palsy. To differentiate PD from DLB, we relied on our time criterium of 12 months in addition to McKeith’s specific criteria (McKeith et al., 2017, 2020). If the disease starts with cognitive impairment or psychiatric symptoms 1 year before, or coincides with beginning motor symptoms, we considered DLB and not PD. However, if motor symptoms preceded either cognitive impairment or psychiatric symptoms, a PD was assumed, and we excluded those patients from our study. Late-onset depression was defined as the first depressive episode occurring after the age of 60 years (Naismith et al., 2012) and late-onset schizophrenia like psychosis was classified as any psychosis appearing after age 40 years (Howard et al., 2000). Our study was conducted in accordance with the latest version of the Declaration of Helsinki, and we obtained approval for this investigation from our local ethics committee of the University Medical Center Göttingen (AZ 10/12/19) before starting the study. Informed consent was obtained from all patients. All methods were carried out in accordance with relevant guidelines and regulations.

The article "Assessing Nigrostriatal Dopaminergic Pathways via 123I-FP-CIT SPECT in Dementia With Lewy Bodies in a Psychiatric Patient Cohort" was published in 2021. Journal: Front Aging Neurosci.

### Statistics

We employed SigmaStat (Version 11, Systat Software GmbH, Düsseldorf) for statistical analysis and SigmaPlot (Version 11, Systat Software GmbH, Düsseldorf) for graph construction. Fisher’s exact test was utilized to compare the frequency of sex, psychiatric features in DLB, psychiatric-onset of DLB, MCI- onset of DLB, one or more core clinical DLB features, core and supportive clinical DLB features, and DLB biomarkers in patients between groups [(1) MCI-onset, psychiatric-onset, mixed-onset of DLB patients as well as (2) patients with a positive 123I-FP-CIT SPECT result compared to those whose 123I-FP-CIT SPECT result was negative] with Bonferroni correction for multiple testing. In addition, the three groups were compared by Student’s *t*-tests were utilized to compare age groups (MCI-onset vs. mixed-onset) and the number of DLB patients (psychiatry cohort, psychiatric features) with possible or probable DLB before and after 123I-FP-CIT SPECT testing over a 6-year period. For not normally distributed group data (psychiatric-onset vs. MCI-onset; psychiatric-onset vs. mixed-onset), we compared the patients’ age *via* the Mann-Whitney *U* test. Fisher’s exact tests were used to compare the number of patients with DLB (psychiatric cohort and psychiatric features) and no LBD after two different classifications (McKeith et al., 2017, 2020) prior to and after their 123I-FP-CIT SPECTs with Bonferroni correction for multiple testing. Furthermore, an ANOVA on ranks was performed for core features, clinical features, supportive biomarkers, and demographics for multiple testing. Furthermore, we did a two factorial ANOVA to analyze the SBR ratio between groups (prodromal DLB, possible DLB, and probable DLB) as one factor and the 123I-FP-CIT SPECT result (no nigrostriatal deficit vs. nigrostriatal deficit) as the other factor. A p-level of <0.05 was considered as significant.

## Results

### Group Categorization

We enrolled 67 patients who had presented in the Department of Psychiatry and Psychotherapy in the UMG with suspected DLB during 2014–2020 and who had undergone 123I-FP-CIT SPECT in the Department of Nuclear Medicine in the UMG. All 67 patients with suspected DLB or probable DLB underwent 123-FP-CIT SPECT. The term suspected DLB entails the following categories: (1) possible DLB, or (2) prodromal DLB patients, or (3) patients with suspected DLB from their neuropsychological examination. Probable DLB patients underwent 123-FP-CIT SPECT with the aim of confirming a probable DLB diagnosis—that is, where we harbored doubts about the diagnosis, or about core clinical features derived from the patient history. Among our 67-patient cohort, we observed positive 123I-FP-CIT SPECT results from 58 patients and negative 123I-FP-CIT-SPECT results from nine patients. We formed three groups categorizing prodromal, possible and probable DLB from those 58 DLB patients presenting a positive nigrostriatal deficit in 123I-FP-CIT-SPECT imaging: (1) with a psychiatric-onset (*n* = 30, psychiatric-onset DLB), (2) MCI-onset (*n* = 15, MCI-onset) or (3) a mixed-onset (mixture of psychiatric and MCI-onset, *n* = 13). Of our patients with a psychiatric-onset and mixed -DLB onset, 18 suffered from late-onset depression and five from a late-onset schizophrenia-like psychosis. At the time of 123I-FP-CIT-SPECT, all patients presented cognitive dysfunction, and parkinsonism was also often present. We classified MCI- and psychiatric-onset DLB patients according to McKeith’s criteria for prodromal DLB (McKeith et al., 2020). The patients with MCI suffered from progressive cognitive impairment. Neither age nor sex differed significantly between these DLB groups (Table 1A). Table 2 shows the numbers of patients with prodromal, possible, and probable DLB before and after 123I-FP-CIT SPECT (Table 2). Among our DLB patients, we differentiated a further subgroup with psychiatric symptoms (anxiety, depression, delusions, apathy) in addition to their neurocognitive impairment (Table 2). Thirty-two of fifty-eight patients (55%) had probable DLB with psychiatric features and a nigrostriatal deficit as verified by 123I-FP-CIT SPECT. MRI was performed in 42 DLB patients (*n* = 24 with a psychiatric-onset, *n* = 7 with an MCI-onset, and in *n* = 11 with mixed-onset); and 14 patients underwent EEG (*n* = 7 with psychiatric-onset, *n* = 2 MCI-onset, and *n* = 5 mixed-DLB onset).

The article "Assessing Nigrostriatal Dopaminergic Pathways via 123I-FP-CIT SPECT in Dementia With Lewy Bodies in a Psychiatric Patient Cohort" was published in 2021. Journal: Front Aging Neurosci.

**TABLE 1A:** Demographic and clinical characteristics of phenotypic differences between DLB patient groups with different clinical onset of symptoms.

	**Psych-onset**	**MCI-onset**	**Mixed onset**	**Statistics psych-**	**Psych- vs.**	**MCI- vs.**	**Comparison of**
	**(*n* = 30)**	**(*n* = 15)**	**(*n* = 13)**	**vs. MCI-onset**	**mixed onset**	**mixed onset**	**three groups ANOVA**
**Demographics**							
Age years	74.6 ± 11.5	77.1 ± 19.8	74.5 ± 20.6	0.25	0.78	0.17^#^	0.52
Sex female N, %	13 (45%)	3 (20%)	5 (38%)	0.28	0.72	0.41	0.31
=1 core clinical feature N, %	17 (57%)	7 (47%)	9 (69%)	0.54	1	0.27	0.39
>1 core clinical feature N, %	6 (20%)	2 (15%)	5 (33%)	0.69	0.19	0.19	0.48
**Main core clinical features**							
Fluctuating cognition N, %	9 (30%)	2 (13%)	4 (31%)	0.28	1	0.37	0.67
REM sleep behavioral disorder N, %	0 (0%)	1 (7%)	0 (0%)	0.33	1	1	0.22
Repetitive hallucinations N, %	11 (37%)	5 (33%)	6 (46%)	0.75	0.73	0.06	0.98
Parkinsonism N, %	18 (60%)	11 (73%)	7 (54%)	0.51	0.74	0.4	0.71
**Supportive clinical features**							
Neuroleptic hypersensitivity N, %	1 (3%)	1 (7%)	2 (15%)	1	0.21	0.21	0.23
Postural instability N, %	5 (17%)	5 (33%)	3 (23%)	0.26	1	0.68	0.89
Repeated falls N, %	3 (10%)	3 (20%)	1 (7%)	0.38	1	0.65	0.68
Syncopes N, %	0 (0%)	0 (0%)	0 (0%)	1	1	1	1
Severe autonomic dysfunction N, %	8 (27%)	1 (7%)	1 (7%)	0.23	0.23	1	0.05
Hypersomnia N, %	0 (0%)	0 (0%)	1 (7%)	1	1	0.46	0.22
Hyposmia N, %	0 (0%)	0 (0%)	2 (15%)	1	1	0.48	0.2
Hallucinations in other modalities N, %	3 (10%)	2 (13%)	4 (31%)	1	0.67	0.05	0.33
Delusions N, %	11 (37%)	1 (7%)	5 (38%)	0.04*	1	0.08	0.08
Apathy N, %	2 (7%)	1 (7%)	1 (7%)	1	1	1	0.96
Anxiety N, %	14 (47%)	1 (7%)	5 (38%)	0.02*	0.74	0.06	0.02
Depression N, %	20 (67%)	4 (27%)	5 (38%)	0.03*	0.1	0.68	0.03
**Supportive biomarker**							
Temporal preservation N, %	6 (20%)	3 (20%)	4 (31%)	1	0.45	0.67	0.66
EEG slowing posterior N, %	1 (3%)	2 (13%)	0 (0%)	0.67	0.25	1	0.12

EEG, electroencephalography, DLB, Dementia with Lewy bodies, MCI, mild cognitive impairment, MCI-onset, mild cognitive impairment onset of symptoms, N, Number, Psych-onset, psychiatric symptom onset, REM, rapid eye movement, SEM, standard error of the mean. Statistics: Fisher’s exact test: *p < 0.05. For comparing age groups a Mann Whitney *U* test was applied, ^#^a student’s test was applied.

The article "Assessing Nigrostriatal Dopaminergic Pathways via 123I-FP-CIT SPECT in Dementia With Lewy Bodies in a Psychiatric Patient Cohort" was published in 2021. Journal: Front Aging Neurosci.

### More DLB Diagnoses *via* 123I-FP-CIT SPECT

If we consider the period between 2014 and 2020, 123I-FP-CIT SPECT does in fact raise the number of probable DLB and probable psychiatric DLB patients significantly (Figures 1A,B, Student’s *t*-test: *p* < 0.05). Furthermore, 123I-FP-CIT SPECT increased significantly the number of patients with prodromal DLB after 123I-FP-CIT SPECT when compared to patients with no DLB, which on the contrary dropped after 123I-FP-CIT SPECT imaging (Figures 2A,B, Fisher’s exact test: *p* < 0.05).

**FIGURE 1:** 123I-FP-CIT-SPECT led to increased numbers of probable DLB patients during 2014–2020. 123-FP-CIT-SPECT led to increased probable DLB patients over a time period of 6 years in our psychiatry cohort **(A)** and in psychiatric-phenotype patients **(B)**. *p < 0.05, student’s *t*-test. DLB was diagnosed twice—before and after the 123-FP-CIT-SPECT.

**FIGURE 2:** Prodromal DLB patients are increased after 123I-FP-CIT SPECT imaging. 123I-FP-CIT SPECT led to increased number of prodromal DLB patients in comparison with non-DLB patients in our psychiatry cohort in **(A)** and in psychiatric-phenotypology patients in **(B)**. *with horizontal line: hereby a significant difference between groups (**A:** number of patients with probable DLB pre-123I-FP-CIT SPECT vs. the number of those with probable DLB post-123-FP-CIT SPECT; **B:** number of patients with probable psychiatric DLB pre-123I-FP-CIT SPECT vs. the number of those with probable psychiatric DLB post-123-FP-CIT SPECT) (*p* < 0.05 Fisher’s exact test) is indicated. DLB was diagnosed twice—before and after the 123-FP-CIT-SPECT.

### Group Comparisons Between DLB Phenotypes

DLB patients (possible and probable) with a psychiatric onset do exhibit a non-significant trend toward a psychiatric-phenotypic appearance more often at stages of full disease manifestation in conjunction with depressive, anxiety, and delusional symptoms than those with a MCI-onset (Table 1A). Other clinical core and supportive features did not differ between these groups. Furthermore, the mixed-onset group did not differ from either the psychiatric-onset or MCI-onset group (Fisher’s exact test, n.s., Table 1A). In addition, an ANOVA on ranks exhibited no significant differences among the three groups (psychiatric-, MCI-, and mixed-onset in DLB patients) in core clinical features, clinical features, and supportive biomarkers (Table 1A). DLB patients with a positive 123I-FP-CIT SPECT revealed a psychiatric-onset of DLB more often than an MCI-onset (Fisher’s exact test, *p* < 0.005).

The article "Assessing Nigrostriatal Dopaminergic Pathways via 123I-FP-CIT SPECT in Dementia With Lewy Bodies in a Psychiatric Patient Cohort" was published in 2021. Journal: Front Aging Neurosci.

### Group Comparisons of Clinical DLB Features in Patients With a Nigrostriatal Deficit to Those Without

We identified no relevant differences between 123I-FP-CIT SPECT -positive and -negative groups in both their core clinical and supportive clinical features (Fisher’s exact test, n.s., Table 1B).

**TABLE 1B:** Characteristics of groups with and without a nigrostriatal dysfunction in 123I-FP-CIT-SPECT.

	**123I-FP-CIT-SPECT+**	**123I-FP-CIT-SPECT-**	**Statistics**
			**Fisher’s exact test value**
**Demographics**			
N of patients LBD	58	9	
Age years (mean ± SEM)	78 ± 0.9	78 ± 2.2	0.073^#^
Sex female n, %	26 (45%)	3 (33%)	0.72
DLB patients with actual psychiatric features n, %	12 (65%)	1 (67%)	0.68
Psych-onset DLB N, %	42 (72%)	4 (44%)	0.12
Delir-onset DLB N, %	1 (2%)	0 (0%)	1
MCI-onset DLB N, %	28 (48%)	6 (67%)	0.47
=1 core clinical feature N, %	13 (57%)	2 (57%)	1
>1 core clinical feature N, %	33 (23%)	5 (22%)	1
**Main core clinical features**			
Fluctuating cognition N, %	12 (21%)	1 (11%)	0.68
REM sleep behavioral disorder N, %	1 (2%)	1 (11%)	0.25
Repetitive hallucinations N, %	18 (31%)	3 (33%)	1
Parkinsonism N, %	36 (62%)	6 (67%)	1
**Supportive clinical features**			
Neuroleptic hypersensitivity N, %	7 (12%)	0 (0%)	0.58
Postural instability N, %	15 (26%)	3 (33%)	0.69
Repeated falls N, %	7 (12%)	1 (11%)	1
Transient episodes of unresponsiveness N, %	0 (0%)	0 (0%)	1
Syncopes N, %	2 (3%)	0 (0%)	1
Severe autonomic dysfunction N, %	11 (19%)	0 (0%)	0.33
Hypersomnia N, %	1 (2%)	0 (0%)	1
Hyposmia N, %	3 (2%)	1 (11%)	0.44
Hallucinations in other modalities N, %	9 (16%)	1 (11%)	1
Delusions N, %	16 (28%)	4 (44%)	0.43
Apathy N, %	4 (7%)	0 (0%)	1
Anxiety N, %	21 (36%)	2 (22%)	0.7
Depression N, %	31 (53%)	6 (67%)	0.72

*LBD, Lewy body dementia, 123I-FP-CIT-SPECT+, 123 I-FP-CIT single photon emission computed tomography with nigrostriatal deficit, 123I-FP-CIT- SPECT-, 123I-FP-CIT single photon emission computed tomography with no nigrostriatal deficit MCI, mild cognitive impairment, N, number, Psych-onset, psychiatric symptom onset, REM, rapid eye movement, SEM, standard error of the mean, Statistics: Fisher’s exact test with the exceptions: ^#^*t*-test.*

The article "Assessing Nigrostriatal Dopaminergic Pathways via 123I-FP-CIT SPECT in Dementia With Lewy Bodies in a Psychiatric Patient Cohort" was published in 2021. Journal: Front Aging Neurosci.

**TABLE 2:** Frequency of DLB types in relation to 123I-FP-CIT SPECT.

	**Prodromal**	**Possible**	**Probable**	**No**
	**DLB**	**DLB**	**DLB**	**DLB**
**Preliminary results, pre 123I-FP CIT SPECT**				
Complete cohort	2	40	13	12
DLB with psychiatric features	1	31	9	8
**Final results, post 123-FP-CIT SPECT**				
Complete cohort	7	16	44	0
DLB with psychiatric features	5	6	32	0

*DLB, dementia with Lewy bodies; 123-FP-CI-SPECT, 123 I-FP-CIT single photon emission computer tomography.*

### Semiquantitative Analysis of 123I-FP-CIT SPECT Between Disease Groups

We conducted a semiquantitative analysis of 123I-FP-CIT SPECT. SBR were calculated in both striata, and the lowest SBR were compared between disease groups (prodromal DLB, possible DLB, and probable DLB) and results from our visual analysis in the entire patient cohort. A two factorial ANOVA revealed no significant group differences in the groups’ SBRs (Figure 3A, ANOVA, n.s.). SBRs were significantly higher in scans of patients who had been visually rated ‘negative’ compared to ‘positive’ scans (ANOVA, *p* < 0.05, Figure 3B).

**FIGURE 3:** Semiquantitative analysis of 123I-FP-CIT-SPECT. Striatum-to-background (SBR) ratios are shown of prodromal, possible, and probable DLB patients in **(A)**. **(B)** Demonstrates significant different SBR ratios between patients with vs. those without a nigrostriatal deficit by visual analysis of 123I-FP-CIT-SPECT. ANOVA: *p < 0.05, n.s., non-significant.

## Discussion

Our main finding is that 123I-FP-CIT SPECT helps us identify more patients presenting probable DLB in a psychiatry cohort and among DLB patients with psychiatric features involving psychotic or affective symptoms. This is the first study to analyze various subtypes of DLB regarding its onset and actual manifestation in a purely psychiatric population. Our second relevant finding is that additional 123I-FP-CIT SPECT imaging is useful when diagnosing prodromal DLB in patients presenting in psychiatric institutions revealing no clear DLB indices before 123I-FP-CIT SPECT imaging. Our results confirm 123I-FP-CIT SPECT’s utility in diagnosing DLB when DLB is suspected but has not yet been diagnosed, or when DLB is diagnosed as being possible—so as to verify the diagnosis of probable DLB. 123I-FP-CIT SPECT seems to be useful not only in those patients with parkinsonism as the cardinal feature, but also in those suffering from visual hallucinations or cognitive fluctuations as core features, indicating the relevance of 123I-FP-CIT SPECT within DLB’s psychiatric and neurocognitive spectrum as observed in psychiatric settings. In addition, 123I-FP-CIT SPECT facilitates the diagnosis of probable DLB and DLB including prodromal DLB in patients presenting a psychiatric phenotype of DLB. We are not in a position to assess REM sleep behavioral disorder as a core feature, as our cohort contained too few patients with REM sleep behavioral disorder and a positive 123I-FP-CIT SPECT result. Another study confirmed such observations, showing that neuropsychiatric symptoms in DLB are more closely related to the extent of functional decline than to any specific symptomology (Borda et al., 2020). Furthermore, our study delivers evidence that 123I-FP-CIT SPECT -positive DLB patients onset more often have a psychiatric-onset (52%), and less often characterized by an MCI-onset of DLB (26%), supporting the relevance of depressive symptoms in suspected DLB patients as the only obvious syndrome at disease onset. Another investigation of a purely psychiatric cohort of 234 patients failed to confirm a relatively high number of DLB patients suffering a psychiatric onset of DLB (Utsumi et al., 2020). However, a clinical caveat is: how can we more accurately distinguish for instance early depressive symptoms due to DLB and those triggered by a major depressive disorder? Obviously, more research is needed into how these disease phenotypologies can be better differentiated. The onset of depressive symptoms might serve as one differentiating criterion, as late-life depressive symptoms can be an early non-neurological sign of either AD or DLB dementia (Thomas et al., 2019). Eighteen patients in our cohort fulfilled this criterion of late-onset depression; five patients presented a late-onset schizophrenia-like psychosis coinciding with an at least psychiatric DLB onset, thus demonstrating the usefulness of lowering the threshold when applying 123I-FP-CIT SPECT in patients not revealing any core clinical features, but who suffer late-onset depression or even a late-onset, schizophrenia-like psychosis. Our study’s additional finding is that the disease’s primary manifestation might be an important factor in its later phenotypic appearance, as more patients with a psychiatric-onset later in disease stage exhibit psychiatric features such as anxiety, depression, and delusions. These findings indicate that psychiatric symptoms are not just important for diagnosing DLB at its onset—they are also relevant in its disease course. Further research is needed to ascertain whether these psychiatric features would benefit from being given more priority when diagnosing DLB, especially in patients demonstrating anxiety, depression, and psychotic symptoms. In particular, delusions or other psychotic symptoms could be more accurately differentiated among disease groups, as a recent study with 350 patients reported a neurodegenerative disorder associated with frequent visual hallucinations [or combined with hallucinations (88%)] compared to major psychiatric disorders (65%) (Schutte et al., 2020). However, most patients diagnosed with a neurodegenerative or major psychiatric disorder exhibited similar psychotic symptoms (Schutte et al., 2020) indicating the need for a biological marker such as 123I-FP-CIT SPECT to better differentiate these disorders, as they share similarities in their phenotypical appearance. The late-onset of a major psychiatric disorder such as late-onset depression might imply a neurodegenerative etiology potentially detectable *via* 123I-FP-CIT SPECT, such as Parkinson’s disease or DLB (Kazmi et al., 2021) especially when other neuroimaging findings are unremarkable. Our results reveal that in DLB patients suffering from psychiatric symptoms, 123I-FP-CIT SPECT plays a key role in diagnosing probable DLB.

The article "Assessing Nigrostriatal Dopaminergic Pathways via 123I-FP-CIT SPECT in Dementia With Lewy Bodies in a Psychiatric Patient Cohort" was published in 2021. Journal: Front Aging Neurosci.

The limitations of our study are: the small size of our patient subgroups restricting the feasibility of drawing practical conclusions, its retrospective character (not assessing DLB criteria and clinical phenomenology at onset and follow up systematically), and that our patient cohort did not contain possible DLB patients exclusively, but rather some with probable DLB also—for whom, although 123I-FP-CIT SPECT can confirm DLB, it is not required to make the diagnosis. Furthermore, as we did not compare our results with a patient cohort from a neurology or movement-disorder clinic undergoing 123I-FP-CIT SPECT, we cannot claim that our results are specific to a psychiatric population. In addition, it is often difficult to know which symptoms patients exhibited when their disease started, in particular when psychiatric or cognitive symptoms coincide. Thus, if no clear differentiation was possible, we assumed a mixed-onset. In addition, the reader should keep in mind when interpreting our findings that DLB is more frequent in a given population if their 123I-FP-CIT SPECT is abnormal. Furthermore, as only some of our DLB patients underwent additional neuroimaging and electroencephalographic examinations, we have no access to other supplemental biomarkers in this retrospective study due to small sample sizes. As limiting factors we must mention due to our study’s retrospective design, that we did not test for anosmia or hyposmia *via* sniffing sticks, and REM sleep behavioral disorder was not confirmed by actual polysomnography in clinical settings for a few patients who exhibited hyposmia and already had a diagnosed REM sleep behavioral disorder (Table 1A). As our findings are not influenced by these low patient numbers, we believe our not having applied these aforementioned methods can be disregarded. However, in future prospective studies these methods should be employed in addition to optimize the clinical phenotyping of DLB patients.

The article "Assessing Nigrostriatal Dopaminergic Pathways via 123I-FP-CIT SPECT in Dementia With Lewy Bodies in a Psychiatric Patient Cohort" was published in 2021. Journal: Front Aging Neurosci.

## Conclusion

In conclusion, 123I-FP-CIT SPECT is an important tool through which to detect decreased striatal dopamine transporter density in patients presenting suspected [appearing as single or multidomain non-amnestic MCI or multidomain amnestic MCI according to McKeith criteria (McKeith et al., 2020)] or possible DLB in a psychiatric cohort or those with psychiatric features. 123I-FP-CIT SPECT helps us diagnose probable and prodromal DLB in patients presenting in psychiatric units. There is evidence of prodromal DLB, namely that 123I-FP-CIT SPECT raises our diagnostic confidence (Thomas et al., 2019), but so far, unfortunately not for those prodromal DLB patients whose onset is psychiatric. Patients with a psychiatric-onset of DLB often at a later disease stage maintain its predominantly psychiatric features. Our retrospective study demonstrates that a large population (55%) of probable DLB patients presenting in psychiatric units displaying a nigrostriatal deficit in 123I-FP-CIT SPECT show a predominant psychiatric phenotypology, indicating that psychiatric DLB seems to be a frequent and underrated subtype of DLB in psychiatric institutions.

## Data Availability Statement

Data are available from the corresponding author.

## Ethics Statement

The studies involving human participants were reviewed and approved by the Ethics Committee of the Medical University Center of Göttingen. Written informed consent for participation was not required for this study in accordance with the national legislation and the institutional requirements.

## Author Contributions

NH and CB wrote the manuscript. NH, CB, CT, and CL designed the study as well as collected and analyzed the data. CB, CL, CT, and JW discussed and revised the manuscript for important intellectual content. All authors contributed to the article and approved the submitted version.

## Conflict of Interest

The authors declare that the research was conducted in the absence of any commercial or financial relationships that could be construed as a potential conflict of interest.

## References

[B1] BallardC. G.JacobyR.Del SerT.KhanM. N.MunozD. G.HolmesC. (2004). Neuropathological substrates of psychiatric symptoms in prospectively studied patients with autopsy-confirmed dementia with lewy bodies. *Am. J. Psychiatry* 161 843–849. 10.1176/appi.ajp.161.5.843 15121649

The article "Assessing Nigrostriatal Dopaminergic Pathways via 123I-FP-CIT SPECT in Dementia With Lewy Bodies in a Psychiatric Patient Cohort" was published in 2021. Journal: Front Aging Neurosci.

[B2] BordaM. G.AarslandD.Tovar-RiosD. A.GiilL. M.BallardC.GonzalezM. C. (2020). Neuropsychiatric Symptoms and Functional Decline in Alzheimer’s Disease and Lewy Body Dementia. *J. Am. Geriatr. Soc.* 68 2257–2263. 10.1111/jgs.16709 32738062

[B3] BrigoF.TurriG.TinazziT. (2015). 123I-FP-CIT SPECT in the differential diagnosis between dementia with Lewy bodies and other dementias. *J. Neurol. Sci.* 359 161–171. 10.1016/j.jns.2015.11.004 26671107

[B4] ChiuP. Y.WangC. W.TsaiC. T.LiS. H.LinC. L.LaiT. J. (2017). Depression in dementia with Lewy bodies: a comparison with Alzheimer’s disease. *PLoS One.* 12:e0179399. 10.1371/journal.pone.0179399 28617831PMC5472293

[B5] CoughlinD. G.IttyerahR.PetersonC.PhillipsJ. S.MillerS.RascovskyK. (2020). Hippocampal subfield pathologic burden in Lewy body diseases vs. Alzheimer’s disease. *Neuropathol. Appl. Neurobiol.* 46, 707–721. 10.1111/nan.12659 32892355PMC7787184

[B6] FujishiroH.OkudaM.IwamotoK.MiyataS.ToriiY.IritaniS. (2018). Early diagnosis of Lewy body disease in patients with late-onset psychiatric disorders using clinical history of rapid eye movement sleep behavior disorder and [(123) I]-metaiodobenzylguanidine cardiac scintigraphy. *Psychiatry Clin. Neurosci.* 72 423–434. 10.1111/pcn.12651 29536584

[B7] Tossici-BoltL.HoffmannS. M. A.KempP. M.MethaR. L.FlemingJ. S. (2006). Quantification of [123I]FP-CIT SPECT brain images: an accurate technique for measurement of the specific binding ratio. *Eur. J. Nucl. Med. Mol. Imaging* 33 1491–1499. 10.1007/s00259-006-0155-x 16858570

[B8] HowardR.RabinsP. V.SeemanM. V.JesteD. V. (2000). Late-onset schizophrenia and very-late-onset schizophrenia-like psychosis: an international consensus. The International Late-Onset Schizophrenia Group. *Am. J. Psychiatry.* 57 172–178. 10.1176/appi.ajp.157.2.172 10671383

[B9] KazmiH.WalkerZ.BooijJ.KhanF.ShahS.SudreC. H. (2021). Late-onset depression: dopaminergic deficit and clinical features of prodromal Parkinson’s disease: a cross-sectional study. *J. Neurol. Neurosurg. Psychiatry* 92 158–164. 10.1136/jnnp-2020-324266 33268471PMC7841491

[B10] KempP. M.ClydeK.HolmesC. (2011). Impact of 123I-FP-CIT (DaTSCAN) SPECT on the diagnosis and management of patients with dementia with Lewy bodies: a retrospective study. *Nucl. Med. Commun.* 32 298–302. 10.1097/MNM.0b013e328343d4ec 21278615

[B11] McCleeryJ.MorganS.BradleyK. M.Noel-StorrA. H.AnsorgeO.HydeC. (2015). Dopamine transporter imaging for the diagnosis of dementia with Lewy bodies. *Cochrane Database Syst. Rev.* 1:CD010633. 10.1002/14651858.CD010633.pub2 25632881PMC7079709

The article "Assessing Nigrostriatal Dopaminergic Pathways via 123I-FP-CIT SPECT in Dementia With Lewy Bodies in a Psychiatric Patient Cohort" was published in 2021. Journal: Front Aging Neurosci.

[B12] McKeithI. G.BoeveB. F.DicksonD. W.HallidayG.TaylorJ. P.WeintraubD. (2017). Diagnosis and management of dementia with Lewy bodies: fourth consensus report of the DLB Consortium. *Neurology* 89 88–100. 10.1212/WNL.0000000000004058 28592453PMC5496518

[B13] McKeithI. G.FermanT. J.ThomasA. J.BlancF.BoeveB. F.FujishiroH. (2020). Prodromal DLB Diagnostic Study Group. Research criteria for the diagnosis of prodromal dementia with Lewy bodies. *Neurology* 94 743–755. 10.1212/wnl.0000000000009323 32241955PMC7274845

[B14] NaismithS. L.NorrieL. M.MowszowskiL.HickieI. B. (2012). The neurobiology of depression in later-life: clinical, neuropsychological, neuroimaging and pathophysiological features. *Prog. Neurobiol.* 98 99–143. 10.1016/j.pneurobio.2012.05.009 22609700

[B15] PalermoG.CeravoloR. (2019). Molecular Imaging of the Dopamine Transporter. *Cells* 8:872. 10.3390/cells8080872 31405186PMC6721747

[B16] SakaiK.IkedaT.IshidaC.KomaiK.YamadaM. (2019). Delusions and visual hallucinations in a patient with Parkinson’s disease with dementia showing pronounced Lewy body pathology in the nucleus basalis of Meynert. *Neuropathology* 39 319–323. 10.1111/neup.12581 31243794

[B17] SchutteM. J. L.LinszenM. M. J.MarschallT. M.FfytcheD. H.KoopsS.van DellenE. (2020). Hallucinations and other psychotic experiences across diagnoses: a comparison of phenomenological features. *Psychiatry Res.* 292:113314. 10.1016/j.psychres.2020.113314 32731082

[B18] SegersK.BenoitF.MeytsJ. M.SurquinM. (2020). Anxiety symptoms are quantitatively and qualitatively different in dementia with Lewy bodies than in Alzheimer’s disease in the years preceding clinical diagnosis. *Psychogeriatrics* 20 242–246. 10.1111/psyg.12490 31782249

[B19] ThomasA. J.DonaghyP.RobertsG.CollobyS. J.BarnettN. A.PetridesG. (2019). Diagnostic accuracy of dopaminergic imaging in prodromal dementia with Lewy bodies. *Psychol. Med.* 49 396–402. 10.1017/S0033291718000995 29692275PMC6331684

[B20] UtsumiK.FukatsuR.YamadaR.TakamaruY.HaraY.YasumuraS. (2020). Characteristics of initial symptoms and symptoms at diagnosis in probable dementia with Lewy body disease: incidence of symptoms and gender differences. *Psychogeriatrics* 20 737–745. 10.1111/psyg.12586 32743894

[B21] WakisakaY.FurutaA.TanizakiY.KiyoharaY.IidaM.IwakiT. (2003). Age-associated prevalence and risk factors of Lewy body pathology in a general population: the Hisayama study. *Acta Neuropathol.* 106 374–382. 10.1007/s00401-003-0750-x 12904992

[B22] WalkerZ.PossinK. L.BoeveB. F.AarslandD. (2015). Lewy body dementias. *Lancet* 386 1683–1697.2659564210.1016/S0140-6736(15)00462-6PMC5792067

